This article has been retracted.

# Hybrid Endovascular Repair in Aortic Arch Pathologies: A Retrospective Study

**DOI:** 10.3390/ijms11114687

**Published:** 2010-11-18

**Authors:** Xiaohui Ma, Wei Guo, Xiaoping Liu, Tai Yin, Xin Jia, Jiang Xiong, Hongpeng Zhang, Lijun Wang

**Affiliations:** Department of Vascular Surgery, Clinical Division of Surgery, Chinese People Liberation Army (PLA) General Hospital and Postgraduate Medical School. 28 Fuxing Road, Beijing 100853, China; E-Mails: maxhtiger@yahoo.cn (X.M.); xiaopingliubj@163.com (X.L.); taiyinbj@163.com (T.Y.); xinjiabjj@163.com (X.J.); jiangxiongbj@163.com (J.X.); hongpengzhangbj@163.com (H.Z.); lijunwangbj@163.com (L.W.)

**Keywords:** aortic arch, endovascular repair, aneurysm, dissection

## Abstract

The aortic arch presents specific challenges to endovascular repair. Hybrid repair is increasingly evolving as an alternative option for selected patients, and promising initial results have been reported. The aim of this study was to introduce our experiences and evaluate mid-term results of supra aortic transpositions for extended endovascular repair of aortic arch pathologies. From December 2002 to January 2008, 25 patients with thoracic aortic aneurysms and dissections involving the aortic arch were treated with hybrid endovascular treatment in our center. Of the 25 cases, 14 were atherosclerotic thoracic aortic aneurysms and 11 were thoracic aortic dissection. The hybrid repair method included total-arch transpositions (15 cases) or hemi-arch transpositions (10 cases), and endovascular procedures. All hybrid endovascular procedures were completed successfully. Three early residual type-I endoleaks and one type-II endoleak were observed. Stroke occurred in three patients (8%) during the in-hospital stage. The perioperative mortality rate was 4%; one patients died post-operatively from catheter related complications. The average follow-up period was 15 ± 5.8 months (range, 1–41 months). The overall crude survival rate at 15 months was 92% (23/25). During follow-up, new late endoleaks and stent-raft related complications were not observed. One case (4%) developed a unilateral lower limb deficit at 17 days and was readmitted to hospital. In conclusion, the results are encouraging for endovascular aortic arch repair in combination with supra-aortic transposition in high risk cases. Aortic endografting offers good mid-term results. Mid-term results of the hybrid approach in elderly patients with aortic arch pathologies are satisfying.

## 1. Introduction

The conventional surgical repair of thoracic aortic aneurysms and dissections remains a high risk procedure [1,2]. Based on the eight largest recent researches published (with over 40 patients) [3–10], the 30-day stroke/death rate after aortic arch surgical repair is up to 25.6% (mean 17.5%). The introduction of endovascular stent graft technology has reached an evolutionary threshold for the treatment of complex aortic diseases. The aortic arch presents specific challenges to endovascular repair, which mainly arise from the involvement of the supra-aortic branches and the tight inner curve. Inoue *et al.* reported one case of triple-branched stengraft [11] and Chuter and colleagues reported a branched stentgraft to the innominate artery [12,13]. However, these new designs are still at an experimental stage. Hybrid repair, which constitutes a combination of open supra-aortic branch revascularization and endovascular aortic repair, has increasingly evolved as an alternative option for selected patients, and promising initial results have been reported [14–18]. The aim of this study was to introduce our expriences and evaluate mid-term results of supra aortic transpositions for extended endovascular repair of aortic arch pathologies.

## 2. Methods

From December 2002 to January 2008, 25 patients with thoracic aortic aneurysms and dissections involving the aortic arch were treated with hybrid endovascular treatment in our center. Preoperative planning was at the discretion of the operating surgeon and was based upon contrast enhanced CT scanning with 1.5 mm cuts and three-dimensional reconstruction that allowed accurate, centerline measurements of the aorta. As a prerequisite for successful stent-graft placement, a proximal landing zone of at least 1.5 cm along the curvature of the aortic arch was necessary. All patients underwent risk evaluation according to EuroSCORE guidelines [19]. Patients who were not suitable for endografting and those at low risk for surgery were treated by open surgery (three patients during the same period).

The average age of the patients was 71.5 ± 9.9 years (range, from 50 to 83 years), and the ratio (male:female) was 5.5:1. Risk factors of the patients are shown in Table 1. Among 25 cases, 14 (56%) were atherosclerotic thoracic aortic aneurysms, the average length of aneurysms was 242.33 ± 82.34 mm; 11 (44%) were aortic dissection, three (12%) were type A thoracic aortic dissection, 8 (32%) were type B thoracic aortic dissection, of which seven were chronic phase and one was acute phase. The acute phase was defined as within two weeks after symptom onset; the subacute phase as the following two-month period; and the chronic phase as anything thereafter. The interval from onset of type B thoracic aortic dissection to treatment was 2–7 months. The average maximum aortic diameter was 64 ± 11.3 mm. None of the pathologies were a result of trauma.

In order to distinguish from Ishimaru’s anatomical aortic classification [20] using antegrade numbering, we propose a retrograde landing zone classification [21]. This classification is based on pathophysiology and reflects the extension of the disease and case complexity, with respect to the need for transposition. We define four proximal landing zones as seen in Figure 1. An endografting procedure at Zone 3 is an ideal situation and requires no surgical complementary step for both aneurysms and dissections. Starting at Zone 2 requires either coverage or transposition of the left subclavian artery (LSA). If the origin of the left common carotid artery (CCA) (Zone 1) is involved, transposition to the right CCA via a carotido-carotid bypass must be performed. We call this adjunctive procedure a hemiarch transposition. If the disease extends the full length of the aortic arch, requiring coverage of the innominate artery (IA), a bypass to the IA and left CCA is performed through a median sternotomy from the ascending aorta. We refer to this as total-arch transposition (Figure 2). The terminology of hemi-arch and total-arch transposition is used in order to simplify the discussion, thus avoiding repetition of the different bypasses performed.

We performed 15 total-arch transpositions and 10 hemi-arch transpositions. For the total-arch transpositions, the endografts were deployed at a second step: 1 week following the creation of the proximal landing zone. We always used a femoral percutaneous access and an additional percutaneous humeral approach was used in some instances to mark the origin of the native IA and LSA. Carotid and vertebral artery circulation were assessed before operation. During the transposition procedure, the stump pressure was checked before clamping the arch vessels.

Hemi-arch transposition was performed via a vertical 4 cm cervical approach to both CCAs. Then an 8 mm Dacron graft (Braun Unigraft, Melsungen) was implanted between two CCAs in a U shape anterior to the trachea. The strategy of this procedure was to perform an end-to-side anastomosis between the left CCA and the brachiocephalic trunk. Afterwards, an end-to-side anastomosis was performed between the LSA and the already transposed LCCA. Total arch transposition is performed through a median sternotomy. A 12 mm Dacron bifurcated graft (Braun Unigraft, Melsungen) was implanted on the ascending aorta as proximal as possible, using lateral clamping. An 8 mm branch anastomosed end-to-end to the IA, while another 8 mm branch was anastomosed the same way to the right CCA. The proximal stumps of these vessels were clamped during the anastomosis and sutured with a 5/0 prolene (Ethicon, Inc, Somerville, NJ, USA) suture after the bypass was finished in order to reduce the clamping time. Depending on the patient’s anatomy, the graft was passed in front or behind the innominate vein, which can be divided or reconstructed if necessary. The LSA was not bypassed unless the vertebral artery was dominating, since it is often hard to reach through a standard sternotomy. Moreover, a patent LSA may serve as access to the aneurysm, when coiling was necessary to treat a residual type I endoleak. A retrograde type II endoleak will appear only if there was an outflow from the sac, such as created by patent intercostal arteries, which are normally thrombosed. In only one case we observed a type II endoleak that was easily treated by percutaneous occlusion of the LSA (Figure 3). Endoleaks are defined as follows: type I include leaks from the proximal and distal seal zones, type II are secondary to patency of aortic branches (intercostal arteries, lumbars, *etc*.) [22].

Following total-arch transposition, markers (metal clips) were placed at the proximal anastomosis to the arch, to define the proximal extent of the proximal landing zone.

Three different commercially available stent-graft systems were used, as shown in Table 2. Endovascular procedures were performed under general anesthesia. In the majority of patients, a transfemoral approach was chosen. If the diameter of the external iliac artery was not large enough, the common iliac artery was used for arterial access. Stent-graft deployment was routinely performed under hypotonic conditions (systolic pressure < 90 mmHg). We did not use adenosine induced transient cardiac asystole. Endografts were oversized by 20% for aneurysms and 10% for dissections. The distal diameter of the endograft was initially slightly reduced with non-tapered devices. Since this series, we have been treating dissections with a tapered endograft whose 24 mm distal diameter better fits the distal landing zone. Stent-graft related data are shown in Table 3. We avoided using dilatation balloons unless it was necessary due to a residual endoleak. This was especially true for dissections.

Following hospital discharge, patients were regularly contacted either by mail or telephone and they were asked to undergo both CT-scan and plain X-ray examinations at 3 (in case of post-operative residual minor type 1 endoleak), 6, 12, 18 and 24 months post-operatively, and yearly there after. Data such as pre-operative size, patients’ condition, risk factors, and post-operative control information, *etc*., were collected during regular working meetings, and were put together in a single Excel file. We calculated crude rates of survival, neurological complications and endoleaks because the study was not large enough to carry out a life-table analysis.

## 3. Results

### 3.1. Duration of Hospital Stay

#### 3.1.1. Surgical Procedure

All patients recovered uneventfully without any serious neurologic injury after aortic debranching. One patient in the hemi-arch transposition group suffered a minor stroke, but was eventually discharged successfully. In the total arch transposition group, one proximal dissection occurred at the site of lateral clamping, which sealed spontaneously.

#### 3.1.2. Stent-Graft Placement

All endovascular procedures were completed successfully. One worsening minor stroke was observed in the hemi-arch transposition group, while no neurological complication occurred in the group of total arch exclusion. During the deployment, the stent graft had not misplacement. We observed three early residual type-I endoleaks (12%), which were left untreated since they may thrombose spontaneously in the post-operative course. The first residual endoleak thrombosed spontaneously and the second was successfully treated by graft extension. The third was due to an uncovered entry tear in the ascending aorta and would have required total arch transposition, which was rejected by the patient. We also had one type-II endoleak in an aneurysm from LSA, which was successfully coiled after one week. We had no case of early paraplegia.

Stroke occurred in three patients (8%) during the in-hospital stage; one patient had a minor stroke within 48 h due to the occlusion of the left CCA bypass, which was resolved by a cervical carotid-carotid bypass. The perioperative mortality rate was 4%; one patient died post-operatively from catheter related complications: The patient died at three days from multiorgan failure after rupture of the descending of the aorta.

### 3.2. Follow-up Period

The average follow-up period was 15 ± 5.8 months (range from 1–41 months), and all patients adopted follow-up regularly. Three-dimensional CT-scan and X-ray examinations were obtained for all the patients before their discharge to act as control images. The overall crude survival rate at 15 months was 92% (23/25). Another patient with chronic obstructive pulmonary disease (COPD) died three months after the procedure because of acute respiratory failure.

During follow-up, new late endoleaks were not observed. The aneurysmal sac exclusion rate was 100%. The rate of occlusion in thoracic false lumen was 91%, while we observed seven cases (28%) patent abdominal false lumens, of which the maximum aortic diameter was <50 mm. Endograft migration, fracture, and stent-raft related complications such as aorto-esophageal fistula were also not observed. None of the patients had new cerebral neurological adverse events. One case (4%) developed a unilateral lower limb deficit at 17 days and was readmitted to hospital. According to independent neurological assessment, this deficit could be due to medullar ischemia, based on cerebral and medullar MRI findings.

## 4. Discussion

Since the first description of revascularization of the left carotid and sbuclavian artery from the ascending aorta prior to stent grafting, only case reports and small case series have been published [24–30]. No comparative randomized or non-randomized studies of combined open debranching and endovascular procedures with other conventional treatment strategies for aortic arch repair have been identified. Furthermore, mid-term and long-term results are still awaited. Our mid-term results of alternative treatment approaches for aortic arch pathologies are satisfying. This hybrid approach provides safe and effective treatment for patients at high risk for conventional repair.

We recommend additional transposition of LSA when it supplies coronary circulation through the left internal mammary artery, when the contralateral vertebral artery (VA) is stenosed or in a diseased vertabro-basilar system. We also recommend transposing the LSA in association with the left CCA when they are included in the aneurysm, except during total transpositions since the LSA is difficult to reach by median sternotomy. In all other cases, LSA transposition is only required later if the coverage becomes symptomatic. Great vessel transposition appears to be safe. There were no major strokes or deaths related to transposition. There was one early death (4%) after the endovascular step, which was either access or guide-wire related.

In the total arch exclusion group, no immediate neurological complications occurred during either surgical or endovascular steps. On the other hand, in the hemi-arch exclusion group, we observed one major stroke. This may be due to catheter manipulation in front of a patent innominate artery ostium, in a patient with an atherosclerotic aorta. A possible way to reduce embolic complications may be to perform pre-operative trans-esophageal echography to better select the patients. We should also pay attention to reduce cross-clamping times of the brain supplying vessels by as much as possible, and furthermore, the absence of substantial atherosclerotic disease in the wall of the asending aorta in total arch rerouting procedures. Without doubt, the risk of embolism is present in all these procedures and careful manipulation of central vessels as well as minimizing the cross-clamp times, in order to not exceed the ischemic frame of cerebral tissue, is mandatory for success [31].

Total arch transposition allows availability of a longer proximal landing zone, easily reaching 3 cm in length for a better anchoring of the endograft. It also avoids stentgraft deployment within the arch curvature, which may cause endoleaks and migration. In selected cases of conical or larger aortas exceeding 40 mm in diameter, the banding technique may be useful in association with total arch transposition to allow a better proximal landing zone.

We prefer a staged procedure for the following reasons: the operating time is decreased; bleeding volume is lowered; the risk of graft infection may be lowered, since endovascular and imaging manoeuvers are not performed in front of an open chest. Considering our encouraging results, we have decided in our department to extend the use of total arch transposition with acute type A aortic dissection. We are combining the replacement of the ascending aorta with the transposition of the IA to the ascending aortic graft. This allows secondary arch coverage for recalcitrant dissection.

The future of this challenging approach is dependent on whether the endografting technology will be reliable or not [32]. Improvement of stent-grafting is needed in terms of flexibility to improve aortic arch navigation and reduce the embolic risk.

In summary, this study analyzed the mid-term results of endovascular repair of aortic arch aneurysm and dissection. The results are encouraging for endovascular aortic arch repair in combination with supra-aortic transposition in high risk cases. Combined treatment for high risk cases offers as good results as seen for conventional surgery for low risk patients. Aortic endografting offers good mid-term results. The mid-term results of the treatment approach in elderly patients with aortic arch pathologies at high risk are satisfying. Nevertheless, meticulous technique is mandatory in order to avoid diverse complications. Thus, the long-term utility of this technology awaits further investigation, although intermediate-term results are encouraging in high-risk patients.

## Figures and Tables

**Figure 1.** The proximal landing zone classification.

**Figure 2.** The intra-operative view of the implanted endograft (left) and the Angiogram (right) demonstrating the reconstruction of the total-arch transposition.

**Figure 3.** Coiling of the left subclavian artery after total arch repair [23].

**Table 1.** Risk factors in patients.

**Risk factors**	**Number of patients**	**Percentage (%)**
Age over 70	17	68
Severe cardiac impairment: cardiac valvulopathy, previous coronary bypass and/or MI	12	48
Chronic pulmonary disease: (FEV_1_ ≤ 1l)	10	40
Neurological dysfunction	3	12
Surgery on thoracic aorta	7	28

**Table 2.** The relevant characteristics of the three proximal device implants used.

**Device**	**Patients treated, %(n)**	**Proximal bare spring**	**Deployment strategy**
Talent (Medtronic, minneapolis, Minn)	32 (8)	With	pullback
Ankura (Lifetech, Shenzhen, China)	24 (6)	With	pullback
Zenith TX2 (Cook, Bjaeverskov, Denmark)	44 (11)	without	Pullback and then release of trigger wire

**Table 3.** Stent-graft related data.

	**Covered length**	**Proximal diameters**	**Distal diameters**	**Graft number**
aneurysm	280.33 ± 82.34 (184–388)	43.33 ± 2.07	38.00 ± 2.19	2.5 ± 1.05
dissection	223.33 ± 111.01 (113–335)	43.33 ± 2.31	42.00 ± 2.00	2 ± 1
